# Network Pharmacology-Based Analysis of the Potential Biological Mechanisms of Coix Seed against Colorectal Cancer

**DOI:** 10.1155/2022/9261768

**Published:** 2022-10-06

**Authors:** Yi Sun, Peishi Jiang, Hongjie Yang, Zhichun Zhang, Yuanda Zhou, Peng Li, Qingsheng Zeng, Xipeng Zhang

**Affiliations:** Department of Colorectal Surgery, Tianjin Union Medical Center, Tianjin 300121, China

## Abstract

**Objective:**

The aim of this study was to explore the potential biological mechanisms of coix seed in the treatment of colorectal cancer (CRC) based on network pharmacology analysis.

**Methods:**

The active components of coix seed and their potential action targets were retrieved from Traditional Chinese Medicine Systems Pharmacology Database and Analysis Platform(TCMSP). The disease targets related to CRC were obtained from the DisGeNET database. The intersection targets of the drug targets and disease targets were selected, and a component-target-disease network was built using Cytoscape 3.8.0 tool. A global network of the core target protein interactions was constructed using String database. Biological function analysis and pathway enrichment analysis of core targets were conducted to explore the potential.

**Results:**

A total of nine active components were obtained from the TCMSP database corresponding to 37 targets. Further analysis showed that 18 overlapping targets were associated with CRC. Kyoto Encyclopedia of Genes and Genomes (KEGG) enrichment analysis was conducted based on the 18 targets and 11 significantly enriched signaling pathways implicated in CRC were identified.

**Conclusion:**

The multicomponent and multitarget characteristics of coix seed are preliminarily verified, and the potential biological mechanisms of coix seed in the treatment of CRC are predicted, which provides a theoretical basis for the experimental research.

## 1. Introduction

Colorectal cancer (CRC) is one of the common malignant tumors of the digestive tract and comprises colon cancer and rectal cancer. Incidence of CRC has been increasing yearly, and the patients are increasingly younger. Previous studies report that CRC disease is associated with factors such as genetics, lifestyle, and diet [1]. The clinical manifestations of CRC include constipation, bloody stool, abdominal distension, and abdominal pain. The intersection of multiple fields such as bioinformatics, molecular medicine, and genetic engineering technology has resulted in significant breakthroughs in clinical treatment of tumors compared with the traditional treatment methods (such as surgery, chemotherapy, and radiotherapy). Tumor molecular targeting and immunotherapy have revolutionized cancer treatment through targeting of target proteins and regulatory signaling pathways implicated in tumor occurrence and development to enhance therapeutic effect [2]. Significance progress has been achieved in use of traditional Chinese medicine for CRC treatment. The use of traditional Chinese medicine improves patients' clinical symptoms and immunity and prevents the recurrence and metastasis of tumor [3]. Traditional Chinese medicine is used for tumor treatment through use of multiple components that target several protein targets and pathways. Traditional Chinese medicine is characterized by broad anticancer activity and few side effects. A systematic study on the mechanism of action of traditional Chinese medicine can be used to identify potential drug targets for CRC treatment [4]. According to the Compendium of Materia Medica where many homologous drugs of medicine and food are recorded, coix seed is not only a medicine for diuresis and dampness, but also a common cereal. The main active components in coix seed include unsaturated fatty acids, steroids, esters, polysaccharides, and triterpenes [5]. Zhou et al. [6] reported that coix seed alleviates experimental colitis in mice through immunoregulation activity. Jinnouchi et al. [7] indicated that coix seed modulates the function of the human immune system by regulating the intestinal microflora. Zhang et al. [8] reported that coix seed effectively relieves pain in patients with tumors, significantly improving the patients' life quality without causing evident adverse reactions. Chen et al. [9] observed that coix seed inhibits the release of histamines and cytokines and suppresses Akt production. Previous studies show that coix seed is the most commonly used traditional Chinese medicine in conservative treatment of CRC [10]. Changfukang and Kanglaite injection developed from coix seed have therapeutic effects on patients with advanced CRC. The two regimens improve the quality of life, have analgesic effects, and prolong the survival time of CRC patients [11]. Coix seed is commonly used in combination with chemotherapy drugs for CRC treatment. Multiple randomized controlled trials indicate that the combination therapy has a higher therapeutic effect and less side effects compared with use of chemotherapy alone [12]. Several studies in modern medicine have shown that the occurrence and development of CRC are associated with the immune status. Traditional Chinese medicine plays an important role in treatment of CRC through modulation of the immune system [13]. Findings from pharmacological studies show that coix seed has antitumor effects and regulates the function of the immune system [14]. However, the mechanism of action of coix seeds in prevention and treatment of CRC has not been elucidated. Therefore, in this study, the network pharmacology approach was adopted to explore the key active components and the mechanism of action of coix seed in prevention and treatment of CRC. The findings provide a theoretical basis for further elucidating the molecular mechanism of action of coix seed in prevention and treatment of CRC through *in vitro* and *in vivo* studies.

## 2. Materials and Methods

### 2.1. Screening of the Phytochemical Composition of Coix Seed

Data on the phytochemical composition of coix seed were retrieved from the Traditional Chinese Medicine Systems Pharmacology Database and Analysis Platform (TCMSP, https://old.tcmsp-e.com/index.php) [15]. Search field (herb name), search term (coix seed), oral bioavailability (OB ≥30%), and drug likeness (DL ≥0.18) were used as the screening criteria for retrieval of phytochemical profile data and properties of coix seed from the database.

### 2.2. Acquisition of Targets for the Active Compounds in Coix Seeds

The targets for the active components obtained in Section 1.1 were retrieved from the TCMSP database (Select “Related Targets” in TCMSP to obtain the corresponding targets to the active compounds of coix seed). The targets were verified using the UniProt database (Universal Protein Resource, https://www.uniprot.org/). A drug-target network was the established using the UniProt ID.

### 2.3. Acquisition of CRC-Related Targets

The targets implicated in CRC were retrieved from the DisGeNet database (DisGeNET Database, https://www.disgenet.org/) by screening the genes related to CRC disease. Diseases was used as the search field, CRC was used as the search term, and Summary of Gene-Disease Associations was used as the range selection [16]. Comparative analysis was conducted on the information of drug targets related to coix seed and the corresponding CRC disease target to obtain the intersection of component targets and disease targets using Venny 2.1.0 tool (https://bioinfogp.cnb.csic.es/tools/venny/). The core targets where drug targets overlapped with disease targets were selected for subsequent analyses.

### 2.4. Establishment of a Component-Target-Disease Network

A component-target and target-disease network was established using coix seed active compounds, targets related to these active compounds, and disease related targets. The component-target and target-disease network files were imported into Cytoscape 3.8.0 tool to build a component-target-disease network of coix seed.

### 2.5. Establishment of Protein-Protein Interaction (PPI) Network and Topological Analysis

The main targets obtained were imported into the String protein interaction database (String, https://cn.string-db.org/) for protein-protein interaction analysis to explore the role of target proteins in CRC. The protein data were used for construction of a PPI based on the component target-disease target network. Protein-protein interactions with an interaction score ≥0.40 were visualized.

### 2.6. Enrichment Analysis

Based on the *R*-package clusterProfiler, the Gene Ontology (GO) enrichment analysis and Kyoto Encyclopedia of Genes and Genomes (KEGG) pathway enrichment analysis were applied to the target proteins. GO functional analysis was performed to explore the function of genes based on the molecular function (MF), biological process (BP), and cellular components (CC) categories [17].

## 3. Results

### 3.1. Screening of Active Compounds

A total of 38 active components isolated from coix seed were retrieved from the TCM-SP database. Further analysis was conducted and 9 compounds with oral bioavailability (OB) ≥30% and drug likeness (DL) ≥0.18, such as sitosterol-alpha1, sitosterol, and mandenol were selected (Table 1).

### 3.2. Targets Related to the Active Compounds

The targets corresponding to the 9 active compounds were obtained from the TCMSP database. A total of 48 related targets were retrieved, which were verified using the UniProt database to obtain 37 targets and their related information. The target gene information of each component is shown in Table 2. The structural formulae of the selected active compounds are shown in Figure 1.

### 3.3. CRC-Related Targets

A total of 5473 genes related to CRC were retrieved from the GeneCards database. The drug target database of coix seed was compared with the corresponding disease target database of CRC using the Venny 2.1.0 tool. A total of 18 overlapping core targets were selected: PGR, NR3C2, NCOA2, ADH1C, RXRA, NCOA1, PTGS1, SLC6A2, ADRB2, AKR1B1, PLAU, LTA4H, CHRM3, ADRA1A, ADRA1B, GABRA1, CHRNA7, and PTGS2.

### 3.4. Drug-Component-Target-Disease Network

A drug-component-target-disease network was established based on the component targets and the disease targets using Cytoscape 3.8.0 tool. The network comprised 22 nodes with 6 drug components and 18 core targets of diseases (Figure 2).

### 3.5. PPI Network

A PPI network was established which comprised a total of 18 common target proteins in coix seed-CRC, forming 3 network units (Figure 3). The node with the highest interaction score was PGR, which interacted with 5 other targets, followed by PTGS2, NCOA2, and NCOA1, which interacted with 4 target proteins each (Figure 4). These results imply that the targets may be important target proteins in mediating the activity of coix seed in CRC treatment.

### 3.6. GO Functional Enrichment Analysis

GO enrichment analysis was conducted on the 18 common target proteins related to coix seed and CRC disease. Significantly enriched molecular function (MF), cellular component (CC), and biological process (BP) categories were screened with threshold of *P* < 0.05. The top 20 BP, MF, and CC terms screened based on adjusted *P* values were identified (Figures 5–7).

### 3.7. KEGG Pathway Enrichment Analysis

KEGG pathway enrichment analysis was performed based on the 18 common target proteins to identify signaling pathways implicated in the functions of the active compounds in CRC treatment. A total of 11 signal pathways were selected with a threshold of *P* < 0.05 (Figure 8).

## 4. Discussion

Traditional Chinese medicine is a systemic treatment method for inducing the body's immune function and overall disease treatment. Several natural active components and traditional Chinese medicine extracts have been widely used in treatment of tumors and other diseases [28, 29]. The holistic and systematic characteristics of network pharmacology are essential in syndrome differentiation and can be used for understanding the effects of traditional Chinese medicine. In the present study, network pharmacology was used in analysis of potential biological mechanisms of coix seed in the treatment of CRC through construction of a comprehensive network of the compounds and targets of coix seed and of the targets related to CRC disease. The results showed the presence of 6 active components including sitosterol, stigmasterol, CLR, sitosterol-alpha1, mandenol, and 2-monoolein potentially associated with the effect of coix seeds in CRC treatment. Previous studies report that stigmasterol is active against lung cancer, ovarian cell cancer, and endometrial cancer by blocking the proliferation cycle of tumor cells and promoting apoptosis of tumor cells [18–20]. In addition, previous findings indicate that sitosterol has significant antitumor activity [25]. Previous results show that stigmasterol and sitosterol are implicated in the treatment of cancer, which is consistent with the results on the components identified in coix seeds related with CRC treatment in this study. CLR is an essential substance in animal tissue cells. It is involved in the formation of cell membranes. CLR is a raw material for the synthesis of bile acids, vitamin D, and steroid hormones [23, 24]. Sitosterol-alpha1 inhibits fungal growth [21]. Mandenol lowers blood cholesterol levels [22]. Previous results indicate that 2-monoolein compound has weak antibacterial activity against *Staphylococcus aureus* [26]. Only few studies have explored the biological activities of CLR, sitosterol-alpha1, mandenol, and 2-monoolein in the treatment for tumors diseases, thus further studies should be conducted to explore the effects and mechanisms of these compounds.

GO function enrichment analysis and KEGG pathway enrichment analysis showed 18 overlapping targets of coix seed and CRC. RXRA, PGR, and NR3C2 proteins are implicated in steroid hormone receptor activity pathways. GABRA1, CHRM3, and CHRNA7 proteins are involved in neurotransmitter receptor activity. PTGS2 and PTGS1 targets are implicated in prostaglandin-endoperoxide synthase activity. RXRA, CHRNA7, PGR, and ADRB2 are involved in chemical carcinogenesis-receptor activation. This preliminary analysis showed that the biological mechanisms of active components in coix seed are implicated in CRC treatment. The study results in this paper are inconsistent with the findings reported by Yahui et al. [30], which may be attributed to the update of the database and the different methods adopted in the two studies.

Core target proteins corresponding the active compounds in coix seed for CRC treatment including PGR, PTGS2, NCOA2, NCOA1, and CHRNA7 were identified through PPI Network analysis. Previous studies reported a significant correlation between low expression of PGR and poor prognosis of CRC patients [31]. PTGS2 expression level is associated with an increase in tumor recurrence and as decrease in CRC specific survival rate. However, PTGS2 expression level is not associated with overall survival rate in patients with colorectal cancer [32]. NCOA2 is a negative growth regulator gene that represses the Wnt/beta-catenin pathway in colorectal cancer. [33]. NCOA1 is known as the “master regulator” of the steroid hormone receptors: estrogen receptor and androgen receptor, which are implicated in breast cancer progression [34]. Chen et al. [9] reported that coix seeds reduce the release of histamines and cytokines and suppresses Akt production. Shi et al. [14] observed that coix seeds inhibit the expression of NF-k*β*, thereby inhibiting epithelial-mesenchymal transition (EMT) of CRC cells induced by TNF-*α*. Yang et al. [35] reported that coix seeds induce apoptosis of cells by inhibiting PI3K and AKT phosphorylation pathway. The findings in the curent study showed that CHRNA7 was the target of stigmasterol, an active component in coix seeds. Notably, *CHRNA7* gene is implicated in the occurrence of CRC. CHRNA7 is an important protein in Ca2^+^-dependent signaling pathways (such as PKA, PKC, PI3K/AKT, and MAPK). PI3K/AKT plays an essential role in various cell activities such as cell proliferation, apoptosis, metabolism, and survival, which can activate NFk*β*. [9] The current results indicate that CHRNA7-Ca^2+^-PI3K-PIP3-AKT-(MTOR, NFk*β*, BIRC5) is a key target signaling pathway of the activity of active components in coix seed for treatment of CRC. Zhou et al. [6] reported that injection of coix seed oil effectively reduced the pain level of cancer patients. Previous findings and the results of this study indicate that the analgesic mechanism of coix seed active compounds may be associated with targeting of the neuroactive ligand-receptor interaction the signaling pathway.

## 5. Conclusion

Network pharmacology and bioinformatics analyses were used to explore the effect of active compounds in coix seed in treatment of CRC disease. The findings showed that the main mechanism of action of coix seed is the regulation of chemical carcinogenesis-receptor activation pathway, targeting calcium signaling pathway, lipolysis in adipocytes, and cGMP-PKG signaling pathway. The results showed that CHRNA7, PGR, PTGS2, NCOA2, and NCOA1 may be the main targets of the active components in coix seed implicated in CRC treatment. This study provides important information to further understand the interaction mechanisms of active compounds and related targets. In addition, the findings provide a basis for further elucidating the molecular mechanism of traditional Chinese medicine compounds in CRC treatment. Network pharmacology technology only qualitatively predicts drug components and targets, and clear pharmacological effects need to be verified through animal experiments and even clinical trials. Network pharmacological approach has certain limitations, thus the results reported in this study should be further verified through *in vivo* and *in vitro* studies. Studies should be conducted to explore the expression profiles of genes and key targets through reverse transcription-polymerase chain reaction and western blot to further elucidate the mechanism of action of the compounds in coix seed.

## Figures and Tables

**Figure 1:** Molecular structures of the active compounds.

**Figure 2:** Network diagram showing the active components in coix seed and their targets against colorectal cancer (Note: The 6 green ellipses represent the active components, the 18 blue diamond nodes represent the main target nodes, and red rectangles represent the disease targets).

**Figure 3:** PPI Network. (a) Target-protein interaction network of the targets related with coix seed and colorectal cancer (Note: The nodes represent proteins and the edges represent protein-protein interactions). (b) The top 16 hub genes (Note: the color code represents interaction scores).

**Figure 4:** Number of action target-protein interactions of active components in coix seed against colorectal cancer (Note: The numbers represent the number of target proteins interacting with the specific protein).

**Figure 5:** The top 20 BP associated with the major targets of coix seed active components. The *y*-axis shows significantly enriched biological terms of the target genes, and the *x*-axis shows the rich factor of the terms (*P* < 0.05). Rich factor represents the ratio of the number of target genes in a specific biological term to the number of all the annotated genes located in that biological term. A higher Rich factor indicates a higher enrichment level. The size of the dot indicates the number of target genes in the biological term, and the color of the dot represents the different FDR ranges.

**Figure 6:** The top 20 MF terms associated with the main targets of coix seed active components. The *y*-axis shows significantly enriched molecular function terms of the target genes, and the *x*-axis shows the Rich factor (*P* < 0.05). Rich factor represents the ratio of the number of target genes in a specific molecular function term to the number of all annotated genes located in that molecular function term. A higher rich factor indicates a higher enrichment level. The size of the dot indicates the number of target genes in the pathway, and the color of the dot represents the different FDR ranges.

**Figure 7:** CC terms for the main targets of coix seed active compounds. The *y*-axis shows significantly enriched cellular component terms of the target genes, and the *x*-axis shows the Rich factor (*P* < 0.05). Rich factor represents the ratio of the number of target genes in a specific cellular component term to the number of all the annotated genes located in that cellular component term. A higher rich factor indicates a higher enrichment level. The size of the dot indicates the number of target genes in the cellular component term, and the color of the dot denotes the different FDR ranges.

**Figure 8:** Enriched KEGG pathways of the main targets of coix seed active compounds. The *y*-axis shows significantly enriched KEGG pathways associated with the target genes, and the *x*-axis shows the rich factor (*P* < 0.05). The Rich factor indicates the ratio of the number of target genes in a specific pathway to the number of all annotated genes in that pathway. A higher Rich factor indicates a higher enrichment level. The size of the dot indicates the number of target genes in a specific pathway, and the color of the dot denotes the different FDR ranges.

**Table 1:** Properties of the active compounds in coix seed and potential mechanisms.

ID	Compound	OB (%)	DL	Reported mechanisms
MOL000449	Stigmasterol	43.83	0.76	Blocking the proliferation of tumor cells [18–20]
MOL001323	Sitosterol-alpha1	43.28	0.78	Inhibition of fungal growth [21]
MOL001494	Mandenol	42	0.19	Lowering cholesterol [22]
MOL000953	Cholesterol (CLR)	37.87	0.68	A raw material for the synthesis of bile acids, vitamin D, and steroid hormones [23, 24]
MOL000359	Sitosterol	36.91	0.75	Interfering with multiple signaling pathways, including cell cycle and apoptosis [25]
MOL008121	2-Monoolein	34.23	0.29	Inhibits *Staphylococcus aureus* [26]
MOL002882	[(2R)-2,3-dihydroxypropyl] (Z)-octadec-9-enoate	34.13	0.3	—
MOL002372	(6Z,10E,14E,18E)-2,6,10,15,19,23-hexamethyltetracosa-2,6,10,14,18,22-hexaene	33.55	0.42	—
MOL008118	Coixenolide	32.4	0.43	Upregulates the expression of regulatory T cells in mice [27]

**Table 2:** Target genes related to the active compounds in coix seeds.

Compound	Target gene
Sitosterol	PGR, NCOA2, NR3C2
Stigmasterol	PGR, NR3C2, NCOA2, ADH1C, IGHG1, RXRA, NCOA1, PTGS1, PTGS2, ADRA2A, SLC6A2, SLC6A3, ADRB2, AKR1B1, PLAU, LTA4H, MAOB, MAOA, PRKACA, CTRB1, CHRM3, CHRM1, ADRB1, SCN5A, HTR2A, ADRA1A, GABRA3, CHRM2, ADRA1B, GABRA1, CHRNA7
CLR	PGR, NR3C2, NCOA2
Sitosterol- alpha1	PGR, PTGS2, GABRA1, ADH1C , NR3C2
Mandenol	PTGS1, PTGS2, NCOA2
2-Monoolein	NCOA2

## Data Availability

The (Active components and their action targets in coix seed and colorectal cancer related disease targets) data used to support the findings of this study have been deposited in the (data repository of herbal (TCMSP) and database of gene-disease associations (DisGeNET)) repository ([https://old.tcmsp-e.com/tcmsp.php and https://www.disgenet.org/]). License Agreement (TCMSP): TCMSP is made available under the Open Database License: https://opendatacommons.org/licenses/odbl/1.0/. License Agreement (DisGeNET): DisGeNET is made available to users subscribing to it, and is made available under the Creative Commons Attribution-NonCommercial-ShareAlike 4.0 International License (https://creativecommons.org/licenses/by-nc-sa/4.0/).
